The article "Optimized Collagen Extraction Process to Obtain High Purity and Large Quantity of Collagen from Human Perirenal Adipose Tissue" was published in 2022. Journal: Biomed Res Int.

# Optimized Collagen Extraction Process to Obtain High Purity and Large Quantity of Collagen from Human Perirenal Adipose Tissue

**DOI:** 10.1155/2022/3628543

**Published:** 2022-03-31

**Authors:** Eun Hye Lee, So Young Chun, Jun Nyung Lee, Bo Hyun Yoon, Jae-Wook Chung, Man-Hoon Han, Tae Gyun Kwon, Yun-Sok Ha, Bum Soo Kim

**Affiliations:** ^1^Joint Institute for Regenerative Medicine, Kyungpook National University, Daegu, Republic of Korea; ^2^BioMedical Research Institute, Kyungpook National University Hospital, Daegu, Republic of Korea; ^3^Department of Urology, School of Medicine, Kyungpook National University, Daegu, Republic of Korea; ^4^Department of Pathology, School of Medicine, Kyungpook National University, Daegu, Republic of Korea

## Abstract

There is growing interest in human adipose tissue-derived collagen as a replacement for animal origin or synthetic materials. Large amounts of adipose tissues around the kidney are being discarded after kidney surgery; thus, we planned to use this tissue as a potentially ideal source of human collagen. Optimization of the collagen extraction process can contribute to the quality, quantity, supply, and cost of collagen production. To extract highly purified and concentrated collagen from human perirenal adipose tissue, we developed a novel extraction process that is superior to the conventional methods in terms of extraction yield, in vitro cytocompatibility, and physicochemical aspects. The sequence of the process and optimized conditions are as follows: (1) destaining with 0.5% H_2_O_2_ for 1 h at 4°C, (2) noncollagenous proteins elimination with 1.5 M NaOH for 24 h at 4°C, (3) atelocollagen preparation with 1.0% pepsin for 48 h at 25°C, and (4) collagen hydrolysis with 1.0 M NaOH for 10 min at 60°C. The final product showed significantly increased hydroxyproline (355.26 ± 18.71 pg/mL) and glycine (22.752 *μ*g/mL) content than the conventional acetic acid hydrolyzed collagen (164.13 ± 1.11 pg/mL and 0.947 *μ*g/mL, respectively). The lyophilized collagen showed more specific peaks for amides A, B, I, II, and III on FT-IR analysis and showed a further native architecture of collagen fibrils in scanning electron microscope images. Therefore, the optimized process can be an effective protocol for extracting collagen from human perirenal adipose tissue.

## 1. Introduction

Collagen is one of the main components of the extracellular matrix (ECM) and plays a critical role in tissue and organ formation [1]. This material is widely used in medical applications, such as drug delivery systems and tissue engineering [2]. Thus far, in most cases, collagen has been derived from animals, such as cows, pigs, fishes, and jellyfishes. However, the use of these nonhuman-derived collagen materials and their products has been limited owing to xenotransplantation-induced immune response, zoonosis, physiochemical instability, and religious reasons in some regions [3, 4].

The article "Optimized Collagen Extraction Process to Obtain High Purity and Large Quantity of Collagen from Human Perirenal Adipose Tissue" was published in 2022. Journal: Biomed Res Int.

In order to overcome these limitations, researchers have attempted to isolate collagen from human tissues, especially from discarded adipose tissue [1]. Usually, human adipose tissue was obtained from subcutaneous adipose tissue via liposuction [5], a cosmetic surgery that removes excess fat from the tissue. Gradually, the range of fat sources has expanded, and visceral fat has been utilized. Among the visceral fat, for the first time, we reported the effective extraction method of ECM from the human perirenal adipose tissue [6]. Perirenal fat tissues are simultaneously resected during the kidney surgeries, and the resected tissue is disposed as medical waste. The amount of discarded human perirenal adipose tissue is continuously rising owing to the increasing number of kidney donations and kidney cancer. There are two limitations in the use of perirenal adipose tissue, as follows: (1) the perirenal adipose tissue-derived ECM is a complex material composed of materials, such as collagen, fibronectin, vitronectin, and laminin, although collagen is present in the highest proportion [6]. (2) The ratio of ECM components may vary, depending on the individual. These questionable qualities are critical disadvantages for expanding the use of perirenal adipose tissue-derived ECM. For quality assurance, the final product needs to be composes of a single factor, that is, pure collagen. In order to increase the purity, the sequence of collagen extraction should be arranged with logic, and each process needs to be optimized.

Conventionally, collagen was extracted from the adipose tissue using acidic hydrolyzing agents and/or enzyme-assisted methods [1, 7]. However, these collagens contain a lot of noncollagenous proteins; low concentrations of glycine, proline, and hydroxyproline or fiber ends form telocollagen that induces immune responses at in vivo condition [8]. Therefore, we devised a multistep process with optimized conditions to increase the purity of collagen and prepare atelocollagen from human perirenal adipose tissue. The product of this optimized process was analyzed in terms of the extraction yield, in vitro cell compatibility, and physicochemical characters. 

## 2. Methods

After obtaining approval from the Institutional Research Ethics Review Board of the Kyungpook National University Hospital (IRB# KNUH 2019-08-008-002), human perirenal adipose tissue was obtained from healthy donors who had undergone donor nephrectomy at the Kyungpook National University Hospital, Deagu, Korea. Perirenal adipose tissue-derived ECM was obtained as described in our previous report [6]. In brief, the perirenal adipose tissue was dissected and dried. The residual lipid in the tissue was removed with acetone and decellularized with 1% Triton X-100. After confirming complete decellularization, ECM was rinsed with deionized water (DW) and air-dried (Figure 1(a)). The ECM was stored at −20°C before use for collagen extraction.

The article "Optimized Collagen Extraction Process to Obtain High Purity and Large Quantity of Collagen from Human Perirenal Adipose Tissue" was published in 2022. Journal: Biomed Res Int.

Our novel collagen extraction process has been illustrated in Figure 1(b). The steps are as follows: step 1, destaining brown pigment; step 2, elimination of noncollagenous proteins; step 3, production of atelocollagen; and step 4, selection of optimal collagen hydrolyzing agent. The criteria for selecting the conditions are based on tissue morphology, histology, glycine, and hydroxyproline concentrations, and at step 4, further collection of products for cytocompatibility, chemical qualities, and physical properties. The properties of the final product were compared to those of the unprocessed ECM.

### 2.1. Destaining with H_2_O_2_ Pretreatment

To remove brown pigment, the ECM was initially treated with hydrogen peroxide (H_2_O_2_, Sigma–Aldrich, St. Louis, MO, USA) solution with various concentrations (0.1%, 0.3%, 0.5%, and 1.0% in 0.1 M sodium hydroxide, NaOH, pH 10). The ECM (25 mg dry weight) was soaked in 1 mL of each H_2_O_2_ solution and agitated with 300 rpm for 1 h at 4°C. After the treatment, the whitened ECM was thoroughly washed with cold DW until a neutral pH was reached. In order to select an optimum H_2_O_2_ concentration, we assessed the ECM color, total protein quantity (Bradford assay, Thermo Fisher, Waltham, MA, USA), and hydroxyproline concentration (ELISA kit, Thermo Fisher). Further, amino acid analysis was performed; each sample was hydrolyzed in 12 N HCl in vacuo under nitrogen at 110°C for 24 h. The hydrolysates were dried at 80°C for 48 h. The pellet was suspended in 0.02 N HCl, and after vortex and sonication, debris were extracted with 0.45-*μ*m filter. The solution (20 *μ*L) was injected to the amino acid autoanalyzer (Hitachi, Tokyo, Japan). All process was carried with an expert operator. The amino acid contents of the each product were expressed as mg/g. The sample prepared under the selected condition was used for the subsequent analysis.

### 2.2. Noncollagenous Proteins Elimination with NaOH

Thereafter, the whitened ECM was treated with NaOH solution to remove the noncollagenous proteins. For determining the optimal NaOH concentration, 0.1 M, 0.5 M, 1.0 M, and 1.5 M NaOH (Sigma–Aldrich) were prepared. The ECM (100 mg wet weight) was soaked in 1 mL of each solution and agitated with 150 rpm at 4°C for 24 h. The NaOH-treated ECMs were analyzed same as above ways, and then select the optimum NaOH concentration.

The article "Optimized Collagen Extraction Process to Obtain High Purity and Large Quantity of Collagen from Human Perirenal Adipose Tissue" was published in 2022. Journal: Biomed Res Int.

### 2.3. Atelocollagen Preparation with Pepsin

To prepare atelocollagen, pepsin was prepared with 0.5%, 1.0%, 1.5%, and 2.0% (w/w) concentration (Sigma–Aldrich, in 0.5 M acetic acid). The ECM (100 mg wet weight) was treated in 1 mL of pepsin solution for 48 h at 25°C with gentle shaking (150 rpm). The pepsin-treated collagen was analyzed, using the method described above; then, the optimum pepsin concentration was selected.

### 2.4. Selection of Collagen Hydrolyzing Agent

For collagen hydrolysis, acidic or basic (alkaline) hydrolyzing agents were prepared. As acidic hydrolyzing agents, organic acids (0.5 M acetic acid and lactic acid, pH 2.5, Sigma–Aldrich) and inorganic acid (1.0 N HCl, pH 2.0, Sigma–Aldrich) were prepared. As alkaline hydrolyzing agent, NaOH (0.5 M, Sigma–Aldrich) was prepared. The ECM (100 mg wet weight) was soaked in 100 *μ*L of hydrolyzing agent for 1 h at 60°C without stirring to prevent the entanglement of the collagen fibers. After the treatment, the insoluble components were separated via centrifugation at 10,000 rpm for 30 min at 4°C. The collected supernatant was adjusted to pH 7.0 and then analyzed using the above-mentioned method; cytocompatibility was added.

For in vitro cytocompatibility analysis, each hydrolyzed collagen was diluted with DW, and the final concentration was adjusted to 10 *μ*g/mL and filtrated with a low protein binding syringe filter (0.2 *μ*m, cellulose acetate, Tisch Scientific, North Bend, OH, USA). The hydrolyzed collagen was coated to a 24-well plate with 100 *μ*L per well for cell morphology observation and coated to a 96-well plate with 30 *μ*L per well for cell proliferation analysis. Each coating was prepared in triplicate. Thereafter, the plates were air-dried overnight in a laminar flow clean bench. After plate surface drying, each well was rinsed with phosphate-buffered saline (PBS), and the cells were seeded with 1 × 103 per well for the 96-well plate and 1 × 105 cells per well for the 24-well plate. The seeded human adipose-derived stem cells were isolated as per a previously described protocol [9] and cultured in Dulbecco's modified Eagle's medium supplemented with 10% fetal bovine serum and 1% penicillin/streptomycin (P/S, all from Invitrogen, Waltham, MA, USA) at 37°C under 5% CO2 in a humidified atmosphere. The cells were used at four passages. Cell proliferation was analyzed with MTT assay on days 1, 3, 5, and 7. At each time point, the cells were harvested with trypsin-ethylenediaminetetraacetic acid (EDTA) in Ca2+- and Mg2+-free PBS (Invitrogen) and resuspended in growth medium. After gentle pipetting, the 100 *μ*L solution was transferred to a 96-well plate. Thereafter, the optical density was measured at 440 nm with a microplate spectrophotometer (IX81, Olympus, Tokyo, Japan). Cell morphology was also observed on the same day with an inverted microscope (Olympus).

The article "Optimized Collagen Extraction Process to Obtain High Purity and Large Quantity of Collagen from Human Perirenal Adipose Tissue" was published in 2022. Journal: Biomed Res Int.

### 2.5. Comparison with Processed and Crude Collagen

The final product, named “processed,” was then compared with the pretreated “crude” ECM with respect to morphology, histology, total protein quantity, hydroxyproline concentration, amino acid analysis, chemical qualities, and physical characterizations with FTIR spectroscopy and scanning electron microscope (SEM). For chemical analysis of the secondary and the triple helix structure, the hydrolyzed collagens with NaOH and crude ECM were lyophilized, and FTIR spectroscopy was performed using a FTIR spectrometer (EQUINOX 55, Bruker, Ettlingen, Germany). Spectra were acquired at a resolution of 4 cm^−1^, and the measurement range was 4000–650 cm^−1^ (mid-IR region) at RT. Automatic signals were collected in 32 scans at a resolution of 4 cm^−1^ and ratioed against a background spectrum recorded from the clean empty cell. Analysis was performed with the OPUS 3.0 data collection software program (Bruker). The physical structure was examined with SEM (S-4300, Hitachi, Tokyo, Japan). The lyophilized sponges were treated with 2.5% glutaraldehyde for 20 min. After fixation, the samples were rinsed with PBS, dehydrated with series of graded ethanol solutions from 50% to 100%, and freeze-dried under vacuum for 2 d. The samples were then coated with platinum via sputtering, and their internal structure was then observed.

### 2.6. Statistical Analyses

The SPSS software package (version 17.0, SPSS Inc., Chicago, IL, USA) was used for the statistical analyses. One-way analysis of variance was performed using the general linear model-univariate procedure from the SPSS software. Differences between the means were evaluated using Duncan's multiple range tests at a significance level of *p* < 0.05 with the SPSS statistical program.

## 3. Results

### 3.1. Pigment Destaining Efficiency as per the H_2_O_2_ Concentration

For the first step, the ECM was treated with H_2_O_2_ for removing the pigment. When the dried ECM was immersed in the H_2_O_2_ solution, bubbles were produced immediately and decreased gradually. During 1 h of treatment, the ECM color turned white, the tissue volume swelled about 3 times, and the structure became loose. The degree of these morphological changes was dependent on the H_2_O_2_ concentration (Figure 2(a)). The total protein quantity was the highest in the 0.5% H_2_O_2_ group (20.38 ± 0.01 *μ*g/mL), followed by the 0.3% H_2_O_2_, 1.0% H_2_O_2_, and 0.1% H_2_O_2_ groups (15.77 ± 0.04 *μ*g/mL, 13.87 ± 0.01 *μ*g/mL, and 10.90 ± 0.01 *μ*g/mL, respectively) (*p* < 0.01) (Figure 2(b)). The hydroxyproline content showed the same result as that in the total protein analysis. The 0.5% H_2_O_2_ group showed the highest value (116.04 ± 6.69 pg/mL), followed by the 0.3% H_2_O_2_, 1.0% H_2_O_2_, and 0.1% H_2_O_2_ groups (104.95 ± 3.57 pg/mL, 102.73 ± 9.24 pg/mL, and 57.97 ± 3.57 pg/mL, respectively) (Figure 2(b)). In the amino acid analysis, 0.5% treatment also showed the highest concentration of total amino acids (Table 1).

The article "Optimized Collagen Extraction Process to Obtain High Purity and Large Quantity of Collagen from Human Perirenal Adipose Tissue" was published in 2022. Journal: Biomed Res Int.

In the histological observation with H&E staining, the ECM fibers were dyed red and exhibited loose distribution depending on the H_2_O_2_ concentration, and the 0.5% H_2_O_2_ group showed the maximal looseness (Figure 2(c)) that can facilitate reagent penetration for the next steps. The fibers treated with 1.0% H_2_O_2_ appeared as condensed bundles. In pigment observation, the ECM treated with 0.1% H_2_O_2_ appeared as several dark spots (arrow), and the frequency was diminished as per the H_2_O_2_ concentration, showing effective removal of the pigments by H_2_O_2_. Based on these results, the optimal H_2_O_2_ concentration was selected as 0.5%.

### 3.2. Efficiency of Noncollagenous Proteins Elimination as per NaOH Concentration

For the second step, the destained ECM was treated with NaOH to eliminate the noncollagenous proteins. The NaOH-treated ECM exhibited a loose, swelled, and semitransparent morphology (Figure 3(a)). The swelling was increased as per the NaOH concentration, and the 0.5-M NaOH, 1.0-M NaOH, and 1.5-M NaOH groups showed an amorphous shape. The total protein concentration was the lowest in the 1.5-M NaOH group (5.71 ± 0.01 *μ*g/mL) as compared to that in the 0.1-M NaOH, 0.5-M NaOH, and 1.0-M NaOH groups (10.13 ± 0.01 *μ*g/mL, 10.17 ± 0.02 *μ*g/mL, and 11.46 ± 0.01 *μ*g/mL, respectively) (*p* < 0.01) (Figure 3(b)). However, the hydroxyproline contents were inverse; the 1.5-M NaOH group showed the highest value (293.97 ± 6.28 pg/mL), and the 0.1-M NaOH, 0.5-M NaOH, and 1.0-M NaOH groups showed significantly lower values (34.29 ± 4.71 pg/mL, 55.93 ± 3.92 pg/mL, and 100.49 ± 1.02 pg/mL, respectively) (*p* < 0.01) (Figure 3(b)). In the amino acids analysis, 1.5-M NaOH treatment showed a high content of total amino acid concentration; in particular, the glycine content was significantly higher (*p* < 0.01) (Table 2). In histological observation, collagen fibers showed loose distribution as per the NaOH concentration, and the 1.5-M NaOH group showed the loosest structure (Figure 3(c)). Based on these results, 1.5 M was selected as the optimal NaOH concentration.

The article "Optimized Collagen Extraction Process to Obtain High Purity and Large Quantity of Collagen from Human Perirenal Adipose Tissue" was published in 2022. Journal: Biomed Res Int.

### 3.3. Efficiency of Atelocollagen Preparation as per the Pepsin Concentration

For the third step, the collagen was treated with pepsin to prepare atelocollagen. As per the morphological observation, the pepsin-treated collagens exhibited a condensed appearance, and the degree increased as per the pepsin concentration (Figure 4(a)). The amount of total protein for 0.5%, 1.0%, 1.5%, and 2.0% pepsin-treated groups was 19.18 ± 0.00 *μ*g/mL, 14.91 ± 0.01 *μ*g/mL, 14.62 ± 0.01 *μ*g/mL, and 15.83 ± 0.01 *μ*g/mL; the total protein content was similar with 1.0%, 1.5%, and 2.0% pepsin treatment (Figure 4(b)). However, the hydroxyproline content was the highest in the 1.0% pepsin-treated group (89.41 ± 1.70 pg/mL), as compared with the 28.37 ± 0.64 pg/mL, 77.20 ± 3.57 pg/mL, and 78.68 ± 2.94 pg/mL in the 0.5%, 1.5%, and 2.0% pepsin treatment groups, respectively (*p* < 0.01) (Figure 4(b)). In the analysis of the amino acid, 1.0% pepsin treatment showed a significantly higher content for glycine and total amino acids (*p* < 0.01) (Table 3). In histological observation, collagen fibers showed loose distribution, and there was no significant difference in the pattern and density along with the pepsin concentration (Figure 4(c)). Based on the hydroxyproline and glycine contents, 1.0% was selected as the optimal pepsin concentration.

### 3.4. Efficiency of Collagen Hydrolysis as per Hydrolyzing Agents

For the fourth step, the atelocollagen was hydrolyzed to prepare hydrolysate. As per the morphological observation after 2 h of treatment with each hydrolyzing agent, the NaOH group showed a homogeneous white opaque color, and the acid-treated groups showed heterogeneous upper suspension and insoluble sediment (Figure 5(a)). After centrifugation, the NaOH group revealed clearly separated supernatant and insoluble sediment, and the acid-treated groups showed dirty upper and lower insoluble sediments. All the supernatants showed viscosity similar to that of a hydrogel.

The amount of total protein for acetic acid-, lactic acid-, NaOH-, and HCl-treated collagen was 18.72 ± 0.04 *μ*g/mL, 17.64 ± 0.01 *μ*g/mL, 10.09 ± 0.01 *μ*g/mL, and 14.29 ± 0.01 *μ*g/mL, respectively. The remaining protein amount was the lowest in the NaOH-treated collagen (*p* < 0.01) (Figure 5(b)). However, the hydroxyproline content was the highest in the NaOH-treated collagen (103.10 ± 1.11 pg/mL), and the contents for acetic acid, lactic acid, and HCl-treated collagen were 76.46 ± 2.94 pg/mL, 89.78 ± 6.93 pg/mL, and 101.99 ± 1.11 pg/mL, respectably (*p* < 0.05) (Figure 5(b)). In the amino acid analysis, the glycine was only detected in the NaOH-treated collagen, and the total amino acid concentration was the highest in this group (Table 4).

The article "Optimized Collagen Extraction Process to Obtain High Purity and Large Quantity of Collagen from Human Perirenal Adipose Tissue" was published in 2022. Journal: Biomed Res Int.

In the analysis of the in vitro cytocompatibility, the NaOH group showed a relatively low cell attachment on day 1; the attached cell number in the control, acetic acid, lactic acid, NaOH, and HCl groups was 22.5 ± 6.45, 59.0 ± 34.57, 62.27 ± 19.58, 38.82 ± 7.97, and 29.12 ± 3.23, respectively. However, the cell proliferation rate was increased in the NaOH group on days 5 and 7, followed by that in the lactic acid group (Figure 5(c)). These different cell proliferation rates were also different in cell morphology; the NaOH and lactic acid group's cells seemed a fibroblast-like morphology, and other group cells showed expended cell shape (Figure 5(d)). Therefore, based on the high hydroxyproline and glycine contents as well as cytocompatibility, the NaOH solution was selected as an optimum hydrolyzing agent.

### 3.5. Comparison between the Processed Collagen and the Crude ECM

Finally, the collagen extracted using the above optimized process was compared with the crude ECM for morphological, chemical, and physical characterizations. The processed collagen showed a whitened phase without debris after hydrolysis (Figure 6(a)), the hydroxyproline content had doubled (355.26 ± 18.71 pg/mL vs. 164.13 ± 1.11 pg/mL) (Figure 6(b)), and the lyophilized morphology was white with fine powder (Figure 6(c)); in the histological observation with H&E staining, collagen fibers appeared evenly spread without condensed form of bundles or stains (arrow, Figure 6(d)); the glycine content was 22 times higher (22.752 *μ*g/mL vs. 0.947 *μ*g/mL), and the total amino acid quantity was about 8 times increased (79.469 *μ*g/mL vs. 9.114 *μ*g/mL) as compared to the crude ECM (Table 5). In FTIR spectroscopy, the peaks of the processed collagen were more specific than for the crude ECM (Figure 6(e)); the wavenumbers for the amide A band was 3400 cm^−1^, that for the amide B band was 2924 cm^−1^, that for the amide I band was 1,643 cm^−1^, that for the amide II band was 1,588 cm^−1^, and that for the amide III band was 1,247 cm^−1^. The internal morphologies were imaged using SEM. The processed collagen showed a rebuild native architecture of collagen fibrils with thinner fibers (Figure 6(f)).

## 4. Discussion

The color of the final product is an important indicator of the collagen quality, especially, the purity. The crude ECM derived from human perirenal adipose tissue showed a dark brown color, even after the processes of delipidation and decellularization were completed. When dissolving this crude ECM in 0.5-M acetic acid (a very commonly used hydrolyzing agent) [1], the hydrolyzed collagen appeared brown color with lot of debris. This morphology is undesirable in the final product; thus, the technical consideration is necessary for stain removal. Our first strategy for high-purity collagen was that of destaining, a method used commonly in the marine industry [10]. However, thus far, it has never been applied to human adipose tissue. The widely used destaining agent is H_2_O_2_. The mechanism of whitening with H_2_O_2_ involves the generation of active oxygen species, such as superoxide (O_2_ˉ), hydroxyl (HO˙), and perhydroxyl (HO_2_˙) radicals by the dissociation of H_2_O_2_ [11]. This process occurs easily at a high pH 11; thus, we prepared H_2_O_2_ in NaOH solution at pH 10. During destaining, the physiological and chemical properties of the ECM were different as per the H_2_O_2_ concentration. Among 0.1%, 0.3%, 0.5%, and 1.0% H_2_O_2_, the 0.5% H_2_O_2_-treated ECM showed the highest protein yield, hydroxyproline content, amino acids concentration, and suitable morphology with a white color. The hydroxyproline and glycine are the main amino acids composing collagen [12]; the hydroxyl group in hydroxyproline makes the structure of collagen more stable [13], and glycine is the most abundant amino acid in every three amino acid position of collagen [14, 15]. The hydroxyproline content was the highest with 0.5% H_2_O_2_; therefore, we selected this concentration.

The article "Optimized Collagen Extraction Process to Obtain High Purity and Large Quantity of Collagen from Human Perirenal Adipose Tissue" was published in 2022. Journal: Biomed Res Int.

In the second step, the noncollagenous proteins were eliminated with NaOH. The elimination theory was as follows: the NaOH-treated matrix swells amorphously due to loss of cohesion by the breakdown of intermolecular bonds within the proteins [16]. The broken peptide bonds easily convert insoluble proteins into soluble proteins, resulting in increased protein hydrolysis [16]. The increased protein hydrolysis enhances the removal of noncollagenous proteins; however, collagen hydrolysis does not occur well because the triple helical structure is difficult to break [16]. Thus, after NaOH treatment, the triple helical collagen component remains, and it increases the collagen content and purity. Among the 0.1-M, 0.5-M, 1.0-M, and 1.5-M NaOH treatments, the 1.5-M NaOH group showed significantly increased hydroxyproline and glycine contents and the lowest total protein quantity, indicating that the collagen purity is increased by the removal of noncollagenous proteins. Therefore, 1.5 M NaOH was selected as an effective concentration for the removal of noncollagenous proteins.

In the third step, collagen was digested with pepsin to remove the nonhelical region at the end of the collagen. The nonhelix telopeptide region acts as a major antigenic determinant that induces an immune response in vivo, and the unwinding region is thermosensitive, causing collagen degradation and denaturation1; thus, it needs to be removed. Pepsin selectively cleaves the terminal nonhelical regions of collagen by breaking the peptide bonds [17] and induces atelocollagen. For effective digestion of the terminal nonhelical region, we adjusted the pepsin concentration and the pH. The optimal concentration is decided by the ECM's structural complexity, strength, and thickness [18]; thus, we tested the range of 0.5%–2.0% concentration as per a report with characteristics similar to our ECM [19]. The pH was settled to an acidic phase with 0.5 M acetic acid solution because the digestive effect of pepsin is increased in an acidic condition1. The 1.0% pepsin-treated group showed the highest hydroxyproline and glycine contents compared to the other concentrations, indicating that this concentration is optimum to make atelocollagen at the same time, with the highest preservation of collagen.

The article "Optimized Collagen Extraction Process to Obtain High Purity and Large Quantity of Collagen from Human Perirenal Adipose Tissue" was published in 2022. Journal: Biomed Res Int.

For the fourth step, the optimum hydrolyzing agent was selected because collagen has triple helix with covalent crosslinks, and it dissolves very slowly, even in boiling water [20]. For complete collagen dissolution, the hydrolyzing agent type, concentration, pH, temperature, and treated time should be considered [21]. Depending on these conditions, collagen viscosity, solubility, water retention, and emulsification capacity can be changed [22]. The commonly reported condition for human adipose collagen hydrolysis is 0.5 M acetic acid, room temperature, and 24-h treatment [21]. In order to evaluate whether these hydrolysis conditions fit our collagen, we tested this condition and added other hydrolyzing agents, such as organic acid (lactic acid), inorganic acid (hydrochloric acid), and basic (alkali, NaOH) agents. Thus far, alkali hydrolysis for human adipose collagen has not been reported. During the hydrolysis, the collagen tissue was mostly dissolved in each hydrolyzing agent, and the NaOH-treated collagen showed a relatively high viscosity and clear phase. In the amino acid analysis, glycine was only detected in the NaOH-treated group, and the hydroxyproline content was also the highest. Considering that the total protein concentration was the lowest in the NaOH-treated collagen, these high glycine and hydroxyproline contents show the high purity and content of collagen. The cytocompatibility analysis also proved the benefit of the NaOH treatment. This group showed the highest cell proliferation for 7 d of culture, indicating that the collagen hydrolyzed in NaOH provides a better microenvironment for cell adhesion and proliferation than other hydrolyzing agents. In particular, the abundance of glycine and hydroxyproline in the NaO-treated group can provide benefit for cell adhesion because these amino acids interact with an adhesion receptor on the cell surface (integrin *α*2*β*1) [23]. As per the cell morphological comparison, the NaOH- and lactic acid-treated groups showed a similar cell shape, such as spindle and triangular, while acetic acid- and HCl0-treated groups showed a spread shape with frill. These results indicate that NaOH is a more suitable hydrolyzing agent as compared to conventional acetic acid. The alkaline extraction may include the following benefits: most of the collagen is dissolved in an alkaline solution, the procedure is simple and cost effective, sterilization is performed during treatment, and the method is bio-safe for human application [23].

The article "Optimized Collagen Extraction Process to Obtain High Purity and Large Quantity of Collagen from Human Perirenal Adipose Tissue" was published in 2022. Journal: Biomed Res Int.

Finally, the processed collagen was compared to the crude ECM for morphological, chemical, and physical characterizations. The processed collagen showed a white and clean morphology in the hydrolysis and lyophilized phase, significantly higher hydroxyproline and glycine content, and neat fibers; these results fulfill the criteria for high purity and quantity. In FTIR spectroscopy, the peaks of the processed collagen were more specific than those of the crude ECM. FTIR spectroscopy was used to detect the functional groups in the collagen. The specific functional groups were connected to the sequence of amino acids to form an *α* chain of type I collagen and consequently determines secondary and the triple helix structures [24]. These amide groups have typical vibrational modes in the infrared spectrum, and each peak means the following: the amide A indicates N–H group, the amide B indicated CH2, the amide I is related to C=O and secondary structure, and the amide II and III demonstrate the existence of a helical structure. If the molecular order is changed, it will reflect via a shift of peak to lower or higher frequency [18]. The processed collagen showed similar locations of peaks with the reported collagen type 118, suggesting a similar molecular order, intermolecular crosslinks, and helical structure. In the SEM analysis, the processed collagen showed a native architecture of collagen fibrils, a network that can give mechanical strength, present cell adhesion molecules allowing cells to enter the network, and provide expanded surface to cell proliferation [25].

In conclusion, the final product manipulated by pigment destaining with H_2_O_2_, noncollagenous protein elimination with NaOH, atelocollagen preparation with pepsin, and hydrolysis with alkali hydrolyzing agent, showed a clean morphology; significantly increased the hydroxyproline (about 2.16 times), glycine (about 24.02 times), and total amino acid (about 8.72 times) content; and maintained the amides A, B, I, II, and III peaks and collagen fibers with native architecture. Therefore, this optimized process can be an effective protocol for extracting collagen with high purity and quantity from human perirenal adipose tissue.

The article "Optimized Collagen Extraction Process to Obtain High Purity and Large Quantity of Collagen from Human Perirenal Adipose Tissue" was published in 2022. Journal: Biomed Res Int.

## Figures and Tables

**Figure 1:** Perirenal adipose tissue-derived extracellular matrix (a) and a concept of collagen extraction process for high purity and good quantity (b).

**Figure 2:** Pigment destaining efficiency as per the H_2_O_2_ concentration: (a) morphological observation, (b) total protein and hydroxyproline concentration, and (c) histological comparison (arrow, pigments). Data are presented as mean ± standard deviation values. The values with different superscript letters in a column are significantly different (*p* < 0.05). Scale bars, 50 *μ*m.

**Figure 3:** Elimination efficiency of noncollagenous proteins as per the NaOH concentration: (a) morphological observation, (b) total protein and hydroxyproline concentration, and (c) histological comparison. Data are presented as mean ± standard deviation values. The values with different superscript letters in a column are significantly different (*p* < 0.05). Scale bars, 50 *μ*m.

**Figure 4:** Atelocollagen preparation efficiency as per pepsin concentration: (a) morphological observation, (b) total protein and hydroxyproline concentration, and (c) histological comparison. Data are presented as mean ± standard deviation values. The values with different superscript letters in a column are significantly different (*p* < 0.05). Scale bars, 50 *μ*m.

**Figure 5:** Collagen hydrolysis efficiency as per hydrolyzing agent: (a) morphological observation, (b) total protein and hydroxyproline concentration, (c) cell proliferation comparison with MTT assay, and (d) cell morphological comparison. Data are presented as the mean ± standard deviation values. The values with different superscript letters in a column are significantly different (*p* < 0.05). Scale bars, 50 *μ*m. Ctrl, uncoated; 0.5 M acetic acid; coated with collagen hydrated with 0.5 M acetic acid; 0.5 M lactic acid, coated with collagen hydrated with 0.5 M lactic acid; 0.5 M NaOH, coated with collagen hydrated with 0.5 M NaOH; 1.0 N HCl, coated with collagen hydrated with 1.0 N HCl.

**Figure 6:** Comparison of the processed collagen and the crude ECM: (a) hydrolyzed collagen comparison, (b) total protein and hydroxyproline concentration, (c) lyophilized collagen comparison, (d) histological comparison (arrow, pigments), (e) FTIR spectroscopy, and (f) SEM images with the network structure of collagen fibers (magnification, ×400; scale bar, 100 *μ*m). Crude, unprocessed ECM; processed, purified collagen through optimized process. Data are presented as the mean ± standard deviation values. The values with different superscript letters in a column are significantly different (*p* < 0.05). Scale bars, 50 *μ*m.

The article "Optimized Collagen Extraction Process to Obtain High Purity and Large Quantity of Collagen from Human Perirenal Adipose Tissue" was published in 2022. Journal: Biomed Res Int.

**Table 1:** Amino acid analysis of collagen after decoloring with different H_2_O_2_ concentration.

Amino acids	0.1% H_2_O_2_	0.3% H_2_O_2_	0.5% H_2_O_2_	1.0% H_2_O_2_
Aspartic acid	0.254	0.265	0.287	0.296
Threonine	ND	ND	ND	ND
Serine	0.056	0.056	0.070	0.075
Glutamic acid	0.195	0.213	0.210	0.221
*Glycine*	0.409	0.478	0.447	0.447
Alanine	0.224	0.266	0.269	0.266
Cystine	1.430	1.461	1.578	1.633
Valine	0.231	0.235	0.248	0.251
Methionine	0.063	0.068	0.074	0.074
Isoleucine	ND	ND	ND	ND
Leucine	ND	ND	ND	ND
Tyrosine	1.409	1.435	1.795	1.577
Phenylalanine	1.302	1.305	1.455	1.483
Lysine	ND	ND	0.016	0.028
Histidine	ND	ND	ND	ND
Arginine	ND	ND	ND	ND
Proline	ND	ND	ND	ND
Total (*μ*g/mL)	5.573	5.784	6.450	6.351

ND: not detected.

**Table 2:** Amino acid analysis of collagen after noncollagenous protein removal with different NaOH concentrations.

Amino acids	0.1 M NaOH	0.5 M NaOH	1.0 M NaOH	1.5 M NaOH
Aspartic acid	ND	ND	0.196	0.028
Threonine	ND	ND	ND	ND
Serine	ND	0.045	0.052	0.23
Glutamic acid	ND	ND	0.104	ND
*Glycine*	ND	0.104	0.315	1.23
Alanine	ND	ND	0.222	0.316
Cystine	0.641	0.653	1.510	2.18
Valine	ND	ND	0.201	0.554
Methionine	ND	ND	0.050	ND
Isoleucine	ND	ND	ND	ND
Leucine	ND	ND	ND	ND
Tyrosine	ND	ND	1.541	ND
Phenylalanine	ND	0.997	1.210	2.006
Lysine	ND	ND	ND	ND
Histidine	ND	ND	ND	ND
Arginine	ND	ND	ND	ND
Proline	ND	ND	ND	ND
Total (*μ*g/mL)	0.641	1.798	5.401	6.546

ND: not detected.

**Table 3:** Amino acid analysis of collagen after treatment with different concentration of pepsin for atelocollagen preparation.

Amino acids	0.5% pepsin	1.0% pepsin	1.5% pepsin	2.0% pepsin
Aspartic acid	0.014	0.276	0.051	0.071
Threonine	ND	ND	ND	0.025
Serine	ND	0.084	0.029	0.220
Glutamic acid	ND	0.243	0.031	0.262
*Glycine*	ND	0.401	0.031	0.026
Alanine	ND	0.274	0.151	ND
Cystine	0.561	1.548	1.007	1.022
Valine	ND	0.288	0.129	0.193
Methionine	ND	0.072	ND	ND
Isoleucine	ND	ND	ND	ND
Leucine	ND	ND	ND	ND
Tyrosine	ND	1.666	ND	ND
Phenylalanine	1.182	1.450	1.005	0.898
Lysine	ND	0.028	0.024	0.031
Histidine	ND	ND	ND	ND
Arginine	ND	ND	ND	ND
Proline	ND	ND	ND	ND
Total(*μ*g/mL)	1.757	6.329	2.458	2.749

ND: not detected.

**Table 4:** Amino acid analysis of collagen after hydrolysis with several acidic or basic hydrolyzing agents.

Amino acids	Acetic acid	Lactic acid	NaOH	HCl
Aspartic acid	0.08	0.934	0.022	ND
Threonine	ND	ND	0.08525	ND
Serine	ND	ND	0.59575	ND
Glutamic acid	ND	ND	0.02225	ND
*Glycine*	ND	ND	1.593	ND
Alanine	ND	ND	0.2985	ND
Cystine	1.892	1.486	0.5255	1.168
Valine	ND	ND	0.27525	ND
Methionine	ND	ND	0.152	ND
Isoleucine	ND	ND	1.31575	ND
Leucine	ND	ND	ND	ND
Tyrosine	ND	ND	1.202	ND
Phenylalanine	1.706	2.63	0.911	1.992
Lysine	ND	ND	0.247	ND
Histidine	ND	ND	ND	ND
Arginine	ND	ND	0.029	ND
Proline	ND	ND	ND	ND
Total (*μ*g/mL)	3.68	5.05	7.274	3.16

ND: not detected.

The article "Optimized Collagen Extraction Process to Obtain High Purity and Large Quantity of Collagen from Human Perirenal Adipose Tissue" was published in 2022. Journal: Biomed Res Int.

**Table 5:** Amino acid analysis of collagen for a comparison between the crude matrix and processed collagen.

Amino acids	Crude	Processed
Aspartic acid	0.479	0.257
Threonine	ND	ND
Serine	0.088	7.399
Glutamic acid	0.288	2.114
*Glycine*	0.947	22.752
Alanine	0.520	5.411
Cystine	2.055	6.076
Valine	0.376	4.826
Methionine	0.191	2.778
Isoleucine	ND	13.615
Leucine	ND	ND
Tyrosine	2.074	ND
Phenylalanine	1.889	7.953
Lysine	0.154	2.913
Histidine	0.052	0.848
Arginine	ND	0.525
Proline	ND	2.003
Total (*μ*g/mL)	9.114	79.469

ND: not detected.

## Data Availability

Data is available on request from the authors.

## Additional Points

*Impact Statement*. To obtain high purity and quantity of collagen from human perirenal adipose tissue, we optimized the collagen extraction method through (1) destaining with H_2_O_2_, (2) elimination of noncollagenous proteins with NaOH, (3) atelocollagen preparation with pepsin, and (4) hydrolysis with alkali. The obtained collagen showed significantly increased hydroxyproline and glycine content, enhanced cytocompatibility, more specific amides peaks, and further native architecture of collagen fibrils than the crude extracellular matrix.

## References

[1] Kim B. S., Choi J. S., Kim J. D., Yoon H. I., Choi Y. C., Cho Y. W. (2012). Human collagen isolated from adipose tissue. *Biotechnology Progress*.

[2] Wallace D. G., Rosenblatt J. (2003). Collagen gel systems for sustained delivery and tissue engineering. *Advanced Drug Delivery Reviews*.

[3] Nagai T., Suzuki N. (2000). Isolation of collagen from fish waste material—skin, bone and fins. *Food Chemistry*.

[4] Helcke T. (2000). Gelatin, the food technologist’s friend or foe. *International Food Ingredients.*.

[5] Mori S., Kiuchi S., Ouchi A., Hase T., Murase T. (2014). Characteristic expression of extracellular matrix in subcutaneous adipose tissue development and adipogenesis; comparison with visceral adipose tissue. *International Journal of Biological Sciences*.

[6] Chun S. Y., Lee J. N., Ha Y. S. (2021). Optimization of extracellular matrix extraction from human perirenal adipose tissue. *Journal of Biometerial Applications*.

[7] Khong N. M., Yusoff F. M., Jamilah B. (2018). Improved collagen extraction from jellyfish (Acromitus hardenbergi) with increased physical-induced solubilization processes. *Food Chemistry*.

The article "Optimized Collagen Extraction Process to Obtain High Purity and Large Quantity of Collagen from Human Perirenal Adipose Tissue" was published in 2022. Journal: Biomed Res Int.

[8] Lynn A. K., Yannas I. V., Bonfield W. (2004). Antigenicity and immunogenicity of collagen. *Journal of Biomedical Materials Research. Part B, Applied Biomaterials*.

[9] Dubois S. G., Floyd E. Z., Zvonic S. (2008). Isolation of human adipose-derived stem cells from biopsies and liposuction specimens. *Mesenchymal Stem Cells*.

[10] Liu W., Zhang Y., Cui N., Wang T. (2019). Extraction and characterization of pepsin-solubilized collagen from snakehead (Channa argus) skin: effects of hydrogen peroxide pretreatments and pepsin hydrolysis strategies. *Process Biochemistry*.

[11] Aïder M., Martel A.-A., Ferracci J., de Halleux D. (2012). Purification of whole brown flaxseed meal from coloring pigments by treatment in hydrogen peroxide solutions: impact on meal color. *Food and Bioprocess Technology*.

[12] Zaelani B., Safithri M., Tarman K., Setyaningsih I., Meydia (2019). Collagen isolation with acid soluble method from the skin of red snapper (lutjanus sp.). *IOP Publishing*.

[13] Wong D. W. (1989). *Mechanism and Theory in Food Chemistry*.

[14] Szpak P. (2011). Fish bone chemistry and ultrastructure: implications for taphonomy and stable isotope analysis. *Journal of Archaeological Science*.

[15] Alhana A., Suptijah P., Tarman K. (2015). Extraction and characterization of collagen from sea cucumber flesh. *Indonesia*.

[16] Kemp G., Tristram G. (1971). The preparation of an alkali-soluble collagen from demineralized bone. *The Biochemical Journal*.

[17] Sato K., Ebihara T., Adachi E., Kawashima S., Hattori S., Irie S. (2000). Possible involvement of aminotelopeptide in self-assembly and thermal stability of collagen I as revealed by its removal with proteases. *The Journal of Biological Chemistry*.

[18] Sinthusamran S., Benjakul S., Kishimura H. (2013). Comparative study on molecular characteristics of acid soluble collagens from skin and swim bladder of seabass (Lates calcarifer). *Food Chemistry*.

[19] Woo J.-W., Yu S.-J., Cho S.-M., Lee Y.-B., Kim S.-B. (2008). Extraction optimization and properties of collagen from yellowfin tuna (Thunnus albacares) dorsal skin. *Food Hydrocolloids*.

[20] Schrieber R., Gareis H. (2007). *Gelatine Handbook: Theory and Industrial Practice*.

[21] Schmidt M., Dornelles R., Mello R. (2016). Collagen extraction process. *International Food Research Journal*.

[22] Karim A., Bhat R. (2009). Fish gelatin: properties, challenges, and prospects as an alternative to mammalian gelatins. *Food Hydrocolloids*.

[23] Hattori S., Adachi E., Ebihara T., Shirai T., Someki I., Irie S. (1999). Alkali-treated collagen retained the triple helical conformation and the ligand activity for the cell adhesion via *α*2*β*1 integrin. *The Journal of Biochemistry.*.

The article "Optimized Collagen Extraction Process to Obtain High Purity and Large Quantity of Collagen from Human Perirenal Adipose Tissue" was published in 2022. Journal: Biomed Res Int.

[24] Adibzadeh N., Aminzadeh S., Jamili S., Karkhane A. A., Farrokhi N. (2014). Purification and characterization of pepsin-solubilized collagen from skin of sea cucumber Holothuria parva. *Applied Biochemistry and Biotechnology*.

[25] Lee C. H., Singla A., Lee Y. (2001). Biomedical applications of collagen. *International Journal of Pharmaceutics*.

